This article has been retracted.

# Al Kharj diabetic patients’ perception about diabetes mellitus using revised-illness perception questionnaire (IPQ-R)

**DOI:** 10.1186/s12875-018-0713-x

**Published:** 2018-02-02

**Authors:** Sameer Al-Ghamdi, Gulfam Ahmad, Ali Hassan Ali, Nasraddin Bahakim, Salman Alomran, Waleed Alhowikan, Salman Almutairi, Tariq Basalem, Faisal Aljuaid

**Affiliations:** 1 Department of Family Medicine, College of Medicine, Prince Sattam bin Abdulaziz University, Al Kharj, Saudi Arabia; 2 Department of Basic Medical Sciences, College of Medicine, Prince Sattam bin Abdulaziz University, Al Kharj, Saudi Arabia; 3 Department of Anatomy, College of Medicine, Prince Sattam bin Abdulaziz University, Al Kharj, Saudi Arabia; 4 Department of Anatomy, College of Medicine, Alazhar University, Cairo, Egypt; 5 Department of Basic Medical Sciences, College of Medicine, Prince Sattam bin Abdulaziz University, Al Kharj, Saudi Arabia; 6 College of Medicine, Prince Sattam bin Abdulaziz University, Al Kharj, Saudi Arabia

**Keywords:** Diabetes, Illness perceptions, Saudi Arabia

## Abstract

**Background:**

Illness perception questionnaires for various medical conditions have become more useful in recent years. However, very few have addressed this issue for Type 2 diabetes in Saudi Arabia.

**Methods:**

A self-administered questionnaire was distributed to Type 2 diabetic patients attendees of primary health care centers and Al Kharj Military Industries Corporation Hospital in Al Kharj, Saudi Arabia, from November 24th 2016 to April 24th, 2017.

**Results:**

Overall, 383 of the 500 distributed questionnaires were returned, and 187 were males (48.8). Most participants understood that what led to diabetes was hereditary, including diet or eating habits. The Cronbach’s alpha value for identity, timeline (cyclical), and emotional factors were relatively high, showing that these scales had a strong level of internal consistency; it also showed that the timeline (acute/chronic) and treatment control scales were low, thus showing internal consistency of these scales. Cronbach’s value of coherence and consequences scales were low.

**Conclusion:**

Saudis with type 2 diabetes mellitus had appropriate knowledge of their disease. They agreed that diabetes was likely to be permanent and would have major consequences on their lives.

## Background

Diabetes mellitus defined as a chronic disease associated with abnormally high levels of glucose in the blood caused by a defect of insulin secretion [1]. Diabetes mellitus is increasingly becoming a health problem globally as a result of increasing prevalence and associated risk of devastating effects or complications on individual for example premature morbidity, kidney failure, gangrene, and even death due to vascular and heart diseases. Diabetes affects both people and the society at large and it has significant impacts health care systems [1–5]. Furthermore, diabetes mellitus is becoming more prevalent worldwide [6], as it has increased from 4.7% to 8.5% in 2014 [7]; in the Middle East and North Africa, it has reached 9.1% in 2015 [8], while in Saudi Arabia, it was as high as 23.9% in 2013 [9].

Illness perception questionnaires for various medical conditions have become more useful in recent years [10]: they examine perceptions patients have about their disease [11, 12], and look at the name of the disease, symptoms of it, and thoughts about its causes [13]. Some studies have been done with this kind of questionnaire [14–17], with a few for diabetes mellitus as well [6, 18]. However, very few have addressed this issue for Type 2 diabetes in Saudi Arabia.

The aim of this research is to examine a Type 2 diabetic patient’s perception of this disease in Saudi Arabia; it can assist health providers in understanding more about what patients feel about their disease, which can in turn help with treatment and future medical care. It is important for patients to grasp various outcomes in chronic diseases, including quality of life and self-management [10].

## Methods

A cross sectional study was conducted over a 5-month period (November 24th 2016 to April 24th, 2017). The targeted population included all Type 2 diabetic patients in Al Kharj governorate, with the study being conducted in Al Kharj Military Industries Corporation Hospital (AKMICH) along with five other primary health care centers (PHCCs) in Al Kharj. The questionnaire was distributed to a largely representative sample of the target population in order to minimize bias, and was conducted with both male and female Type 2 diabetics who attended PHCCs and AKMICH in Al Kharj governorate.

### Sampling methods and sample size

A multi-stage random cluster sampling technique was employed in the PHCCs, according to their geographic divisions in five districts (middle, northern, southern, western, and eastern) with two to three in each. We randomly chose one PHCC in each district, with five PHCCs in total. Eligibility criteria included being Saudi, having T2DM for at least 1 year, being 18-years-old or more, no cognitive impairment that could interfere with communication or comprehending questions, being able to read and write in Arabic, having no visual impairment that could interfere with self-reporting, and willingness to participate in the study. Extremely ill patients and pregnant women were not eligible.

Given that the prevalence of diabetes mellitus in Saudi Arabia is 23.9%, and the total population of Al Kharj governorate is 376,325 [19], the minimum sample size required for a 99% confidence interval (CI) with a 5% margin of error was calculated to be 383. The sample size was adjusted to 400 to account for any possible data loss during collection. To compensate for low response and rejection due to non-eligibility, 25% was added as well. Thus, the target sample size was 500. The flow chart shows the data collection process with the response rate (as shown in Fig. 1).

**Fig. 1:** Data Collection Process Flowchart

### Data collection instrument

A validated, multiple selection, self-administered illness perception questionnaire (IPQ-R) was used as the data collection tool, which was established at University I Bergen. It was used with the permission to assess diabetes illness perceptions, with a version for diabetes available on their website [20].

The illness perception questionnaire was translated into Arabic, reviewed by Family Medicine consultants, and then translated back into English. The questionnaire contained a total of 85 questions, with 84 close-ended questions and 1 open-ended question. A pilot study of 30 participants was done before distribution of the questionnaire at no change: participants did not face any difficulties filling it out. Demographic data about participants (age, gender, education level, occupation, marital status, other chronic diseases, type of treatment [either insulin or tablet], and duration of diabetes) were obtained.

### Data entry and analysis

Statistical Package for Social Sciences (SPSS) software version 23 was used for data entry and analysis where descriptive statistics where frequencies, percentages, mean and standard deviation will be used to measure the central tendency and distribution of the variables. T-test analysis were also conducted.

In addition, Subgroup analyses were also conducted to determine the illness perceptions among patients. This will help in understanding the participant’s perception on how the illness change with disease progression (e.g. type of treatment, complications, etc.).

### Ethical consideration

Letters of authorization were obtained from each hospital before distribution, with verbal informed consent from participants. Hard copies of the translated questionnaire were stored in the main hospital and five primary health care centers in Al Kharj governorate.

## Results

The youngest study participant was 18-years-old, while the oldest participant was 85-years-old, with most participants between 30 and 70 years of age: age distribution was not skewed. The mean age (M = 46.0, SD = 15.94) showed that the sample was middle age on average.

The minimum time period in which participants lived with diabetes was one year, while the maximum time period was 40 years. The duration was skewed with a few participants having lived with it for more than 20 years, although the median duration was 6 years. The number of study participants on oral hypoglycemic agents (OHA) was higher than those on insulin, with or without OHA. More than half of the study participants were unemployed, while those who did not have a chronic disease was higher than those with only one. Those who were educated were significantly greater than those who were not, with results shown in Table 1.

**Table 1:** Sociodemographic characteristics and disease profile (*n* = 383)

		N	%
Gender	Male	187	48.8
	Female	196	51.2
Diabetes medication	OHA	220	57.4
	Insulin with or without OHA	163	42.6
Chronic diseases	No	218	56.9
	Yes	165	43.1
Education	Educated	308	80.4
	Not educated	75	19.6
Marital status	Single	117	30.5
	Married	266	69.5
Employment status	Employed	186	48.6
	Unemployed	197	51.4

A Student’s t-test showed the mean duration between male and female participants was not statistically different. Unemployed study participants demonstrated a higher mean duration compared to employed participants, with a t-test showing this difference to be statistically significant. Study participants who were on insulin, with or without OHA, had a higher mean duration compared to participants who were on OHA, with a t-test showing this difference to be statistically significant as well. Participants with a chronic disease had a longer duration compared to participants who did not have one, with a t-test revealing this difference to be statistically significant. Moreover, participants who were not educated also had it for a longer time period compared to those who were educated, with a t-test showing the difference to be statistically significant as well.

The shortest time period for having diabetes among participants was 31–45 years: those over 61 years had it for a longer duration. A one-way analysis of variance (ANOVA) was used if the mean in age categories was significantly different, as it also showed that the mean in age categories was statistically different [F (4,378) = 28.13, *p* = 0.000].

The descriptive statistics and Chi-square results of each symptom, along with the belief that the symptom was associated with diabetes are shown in Table 2. Chi-square tests were used if there was any association between symptoms, or the belief that it was associated with diabetes, as the test showed an association with some symptoms. These symptoms included loss of strength, dizziness, sleep difficulties, upset stomach, stiff joints, weight loss, and nausea.

**Table 2:** The association between experience any symptom since diabetes and believe that these symptom is related to diabetes

Symptom		Belief symptom is related to diabetes			
		No	Yes	χ	p
1. 1. Pain	Yes	201 (61.1%)	50 (58.8%)	0.146	0.70
	No	128 (38.9%)	35 (41.2%)		
2. 1. Sore throat	Yes	261 (67.3%)	16 (61.5%)	0.361	0.55
	No	127 (32.7%)	10 (38.5%)		
3. 1. Fatigue	Yes	128 (67.4%)	165 (73.7%)	1.97	0.161
	No	62 (32.6%)	59 (26.3%)		
4. 1. Nausea	Yes	176 (50.6%)	48 (72.7%)	10.96	0.001^*^
	No	172 (49.4%)	18 (27.3%)		
5. 1. Breathlessness	Yes	171 (45.7%)	22 (55.0%)	1.25	0.318
	No	203 (54.3%)	18 (45.0%)		
6. 1. Weight loss	Yes	84 (48.6%)	146 (60.6%)	5.89	0.015^*^
	No	89 (51.4%)	95 (39.4%)		
7. 1. Fatigue	Yes	128 (67.4%)	165 (73.7%)	1.97	0.161
	No	62 (32.6%)	59 (26.3%)		
8. 1. Stiff joints	Yes	163 (48.2%)	51 (67.1%)	8.86	0.003^*^
	No	175 (51.8%)	25 (32.9%)		
9. 1. Sore eyes	Yes	156 (45.3%)	40 (57.1%)	3.25	0.072
	No	188 (54.7%)	30 (42.9%)		
10. 1. Wheeziness	Yes	175 (47.4%)	24 (53.3%)	0.561	0.454
	No	194 (52.6%)	21 (46.7%)		
11. 1. Headaches	Yes	149 (60.8%)	108 (63.9%)	0.41	0.524
	No	96 (39.2%)	61 (36.1%)		
12. 1. Upset stomach	Yes	111 (39.9%)	75 (55.1%)	8.55	0.003^*^
	No	167 (60.1%)	61 (44.9%)		
13. 1. Sleep difficulties	Yes	125 (42.2%)	67 (56.8%)	7.18	0.007^*^
	No	171 (57.8%)	51 (43.2%)		
14. 1. Dizziness	Yes	50 (36.5%)	168 (60.6%)	21.45	0.000^*^
	No	87 (63.5%)	109 (39.4%)		
15. Loss of strength	Yes	40 (26.7%)	114 (43.2%)	11.17	0.001^*^
	No	110 (73.3%)	150 (56.8%)		

Table 3 shows that most participants believe there is a lot they can do to control symptoms, what they do can determine whether diabetes gets better or worse and the course of diabetes depends on them. Almost two third of participant believe they have the power to influence diabetes, there is very little that can be done to improve diabetes and treatment can control diabetes.

**Table 3:** Participants views about diabetes (n = 383)

Views about diabetes	Strongly agree or agree
	Percent (%)
My diabetes will last a short time	24.5
My diabetes is likely to be permanent rather than temporary	60.3
My diabetes will last for a long time	51.4
This diabetes will pass quickly	12.5
I expect to have this diabetes for the rest of my life	59.0
My diabetes is a serious condition	53.3
My diabetes has major consequences on my life	65.3
My diabetes does not have much effect on my life	25.3
My diabetes strongly affects the way others see me	36.8
My diabetes has serious financial consequences	40.2
My diabetes causes difficulties for those who are close to me	44.9
There is a lot which I can do to control my symptoms	80.4
What I do can determine whether my diabetes gets better or worse	80.2
The course of my diabetes depends on me	80.4
Nothing I do will affect my diabetes	21.9
I have the power to influence my diabetes	72.6
My actions will have no effect on the outcome of my diabetes	23.5
My diabetes will improve in time	43.9
There is very little that can be done to improve my diabetes	77.8
My treatment will be effective in curing my diabetes	22.7
The negative effects of my diabetes can be prevented (avoided) by my treatment	76.0
My treatment can control my diabetes	77.5
There is nothing which can help my condition	13.6
The symptoms of my condition are puzzling to me	42.0
My diabetes is a mystery to me	23.0
I don’t understand my diabetes	32.4
My diabetes doesn’t make any sense to me	33.4
I have a clear picture or understanding of my condition	16.7
The symptoms of my diabetes change a great deal from day to day	57.7
My symptoms come and go in cycles	62.9
My diabetes is very unpredictable	59.5
I go through cycles in which my diabetes gets better and worse.	77.3
I get depressed when I think about my diabetes	42.8
When I think about my diabetes I get upset	49.6
My diabetes makes me feel angry	29.2
My diabetes does not worry me	43.9
Having this diabetes makes me feel anxious	54.0
My diabetes makes me feel afraid	42.6

More participants understood that what led to diabetes was hereditary, including diet or eating habits. There was fair agreement that aging, behavior, poor medical care in the past, as well as stress or worry also contributed. Other causes had a low level of agreement, as shown in Table 4.

**Table 4:** Diabetes cause perceptions (n = 383)

Cause	Strongly agree or agree
	Percent (%)
Stress or worry	40.5
Hereditary - it runs in my family	75.5
A Germ or virus	19.8
Diet or eating habits	62.4
Chance or bad luck	26.9
Poor medical care in my past	39.9
Pollution in the environment	12.3
My own behavior	43.9
My mental attitude e.g. thinking about life negatively	23.0
Family problems or worries	25.3
Overwork	28.5
My emotional state e.g. feeling down, lonely, anxious, empty	23.0
Ageing	46.7
Alcohol	13.3
Smoking	15.1
Accident or injury	8.4
My personality	20.6
Altered immunity	19.3

The Cronbach’s alpha value for identity, timeline (cyclical), and emotional factors were relatively high, showing that these scales had a strong level of internal consistency; it also showed that the timeline (acute/chronic) and treatment control scales were low, thus showing internal consistency of these scales. Cronbach’s value of coherence and consequences scales were low, showing a moderate level of internal consistency, as seen in Table 5.

**Table 5:** Diabetes illness perceptions based on the Revised Illness Perception Questionnaire (IPQ-R) scale

IPQ-R	Number of items	Possible score range	Mean (SD)	Cronbach’s alpha
Identity	14	0–16	4.42 (3.57)	0.87
Timeline (acute/chronic)	6	6–30	18.14 (2.60)	0.19
Timeline (Cyclical)	4	4–20	13.30 (2.96)	0.74
Consequences	6	6–30	17.22 (3.58)	0.50
Personal control	6	6–30	19.28 (2.71)	0.41
Treatment control	5	5–25	15.51 (2.16)	0.22
Emotional	6	6–30	16.03 (4.37)	0.61
Coherence	5	5–25	12.75 (3.42)	0.54

## Discussion

The study drew its sample across the age spectrum of the population, with the youngest participant aged 18 and the oldest participant aged 85. Therefore, the possibility of age bias was minimized, as findings were generalizable across an age spectrum of the population. The percent of male participants was 48.8 and female participants was 51.2, which was fairly balance, such that the risk of too many participants from one gender was minimized. Due to an equitable distribution between genders, the findings could be generalized across genders. To further minimize risk of bias in the sample population, study participants were carefully selected to ensure educational, marital, and employment status.

We did not find a significant difference in how long male or female participants had lived with diabetes. Although this suggests similarity in its occurrence among men and women, it cannot be concluded that risk factors are similar. More research is needed to characterize this issue.

Study participants with chronic diseases had lived for a significantly longer time period with diabetes, compared to study participants without chronic disease. One possible explanation of this finding is that diabetes is associated with other diseases. Therefore, people with other diseases were at higher risk of developing diabetes at an earlier age. The Centers for Disease Control and Prevention reported that those 45–64 years had the highest risk of developing diabetes [21], but that lifestyle risk had also placed a younger population at high risk of developing diabetes. Due to this variation in environmental factors, more research is required to understand high risk factors in the population.

Uneducated participants had lived with diabetes for a significantly longer period than educated participants, although it is difficult to delineate the main cause of this difference (whether due to income, lifestyle, or quality of life between employed and unemployed populations). For example, Eva et al. studied factors associated with knowledge of diabetes in patients with a higher level of education than those without one [22]. Furthermore, Michell et al. found that only 10.8% knew that diabetes could be prevented [23]. More research is similarly required to understand relevant differences in risk factors because of the huge burden of diabetes management on families and healthcare systems [24].

Although diabetes had been associated with older populations, this study found it in younger populations as well, despite that older populations had lived with it for a longer time period. This study found that after 60 years of having lived with diabetes, it was more than double than those aged 45 years or less who had lived with it. Due to the high economic and social costs of managing diabetes, more studies are needed in the younger population to understand and mitigate its risk factors.

Participants associated loss of strength, dizziness, sleep difficulties, upset stomach, stiff joints, weight loss, and nausea with diabetes. The questionnaire was designed to be targeted toward the cognitive representations of the five components of the disease (diabetes). The study participants were asked about their cognitive representations of the five components of the diabetes. From the study results, some participants (patients) had an inadequate level of knowledge of diabetes management. Therefore, there is need to introduce education program to educate patients on how to identify and manage symptoms. The education program will also help the patients to have a good understanding of diabetes because and to identify the most probable causes of diabetes.

### Study findings

Based on the study findings, it was found that the two causes patients had a high level of agreement they were linked to diabetes were eating habits and hereditary. Knowledge of diabetes was good because patient views on diabetes were consistent with reality. More patients agreed diabetes was likely to be permanent as opposed to lasting for a short time. This is in line with findings of Michell et al. who found slightly more than half of their study participants knew they would not be cured of diabetes [23]. More patients agreed diabetes had major consequences on their life and they could put an effort towards managing diabetes. This finding was consistent with the results of a study by Fatma, Mohamed, Juma and Bachar who found in the UAE patients had a positive attitude to self-care. Successfully managing diabetes was possible because this study found there were patients who had lived with diabetes for more than 20 years [25].

## Conclusion

Based on the study results, diabetes mellitus and high risk patients reported knowledge and attitudes conducive to good health; however, the majority of the participants did not translate these positive traits into healthy behavior with respect to weight loss, exercise and nutrition or diet.

The study results indicated that some participants (patients) had an inadequate level of knowledge of diabetes management. Therefore, there is need to introduce education program to educate patients on how to identify and manage symptoms. The education program will help the patients to have a good understanding of diabetes because and to identify the most probable causes of diabetes.

It is clear that there is a need to adopt early and intensive interventions in Al Kharj diabetic patients or people diagnosed with the disease since this will help in reducing the risks of disease progression as well as minimize the risk of microvascular and microvascular complications or other complications related to the disease. There is also the need to improve the delivery of health care to individuals with chronic conditions and reduce any barriers to the early utilization of insulin.

In conclusion, the problem of diabetes mellitus on the health care system calls for efforts to more optimally treat diabetic patients and to prevent the development of diabetes development in individuals at risk.

### Implications of the study

The study provides an in-depth and comprehensive perception and knowledge of Al Kharj diabetic patients about their illness using Revised-Illness Perception Questionnaire (R-IPQ). Based on the study findings, the study also proposes clear recommendations for improving management and prevention of diabetes in Al Kharj. The study will help in developing policies and programs for better cost effective strategies of diabetes treatment and prevention methods as well as effective management of diabetes and cost effective strategies in Al Kharj and the health care setting in general. This research will benefit diabetic patients by generating evidence based strategies that can be used in formulating policies and programs targeting the general diabetic patients to help them manage the illness.

### Recommendations

The study made the following recommendations:

- Optimize the use of therapies that are presently available to reduce complications and ensure sufficient glycemic, blood pressure, as well as proper lipid control.
- Improve Al Kharj diabetic patients adherence to pharmacologic and lifestyle interventions.
- Educate the patients on diabetes self-management
- The study recommends that Al Kharj diabetic patients need to change their lifestyle habits i.e. change eating habits and increase exercise.
- The study recommends that health literacy programs be adopted in health care facilities and clinics.
- The study recommends formulation of programs and policies and targeting the general diabetic patients to help them manage the illness.

## Abbreviations

AKMICH: Al Kharj Military Industries Corporation Hospital
CI: Confidence interval
IPQ-R: Revised Illness Perception Questionnaire
M: Mean
OHA: Oral Hypoglycemic Agents
PHCCs: Primary Health Care Centers
SD: Standard Deviation
SPSS: Statistical Package for Social Sciences
T2DM: Type 2 Diabetes Mellitus
